The article "High-Resolution Computer Tomography Image Features of Lungs for Patients with Type 2 Diabetes under the Faster-Region Recurrent Convolutional Neural Network Algorithm" was retracted in 2023. Reasons: signs of a paper mill; suspected computer-generated content; unreliable results or conclusions; concerns about the data.

# High-Resolution Computer Tomography Image Features of Lungs for Patients with Type 2 Diabetes under the Faster-Region Recurrent Convolutional Neural Network Algorithm

**DOI:** 10.1155/2022/4147365

**Published:** 2022-04-25

**Authors:** Yumei He, Juan Tan, Xiuping Han

**Affiliations:** ^1^Department of General Medicine, Affiliated Hospital of Yan'an University, Yan'an, 716000 Shaanxi, China; ^2^Department of Traditional Chinese Medicine, Affiliated Hospital of Yan'an University, Yan'an, 716000 Shaanxi, China

## Abstract

The objective of this study was to adopt the high-resolution computed tomography (HRCT) technology based on the faster-region recurrent convolutional neural network (Faster-RCNN) algorithm to evaluate the lung infection in patients with type 2 diabetes, so as to analyze the application value of imaging features in the assessment of pulmonary disease in type 2 diabetes. In this study, 176 patients with type 2 diabetes were selected as the research objects, and they were divided into different groups based on gender, course of disease, age, glycosylated hemoglobin level (HbA1c), 2 h C peptide (2 h C-P) after meal, fasting C peptide (FC-P), and complications. The research objects were performed with HRCT scan, and the Faster-RCNN algorithm model was built to obtain the imaging features. The relationships between HRCT imaging features and 2 h C-P, FC-P, HbA1c, gender, course of disease, age, and complications were analyzed comprehensively. The results showed that there were no significant differences in HRCT scores between male and female patients, patients of various ages, and patients with different HbA1c contents (*P* > 0.05). As the course of disease and complications increased, HRCT scores of patients increased obviously (*P* < 0.05). The HRCT score decreased dramatically with the increase in the contents of 2 h C-P and FC-P after the meal (*P* < 0.05). In addition, the results of the Spearman rank correlation analysis showed that the course of disease and complications were positively correlated with the HRCT scores, while the 2 h C-P and FC-P levels after meal were negatively correlated with the HRCT scores. The receiver operating curve (ROC) showed that the accuracy, specificity, and sensitivity of HRCT imaging based on Faster-RCNN algorithm were 90.12%, 90.43%, and 83.64%, respectively, in diagnosing lung infection of patients with type 2 diabetes. In summary, the HRCT imaging features based on the Faster-RCNN algorithm can provide effective reference information for the diagnosis and condition assessment of lung infection in patients with type 2 diabetes.

## 1. Introduction

Diabetes is a chronic metabolic disease caused by the inability of the human body to produce insulin or the insulin produced cannot be utilized by the human body [1]. As a hormone that regulates blood sugar, insulin will increase blood sugar in diabetic patients when it fails to perform its normal function, and its long-term existence will cause serious damage to the blood vessels and nerves [2, 3]. Diabetes can be divided into two types. Type 1 diabetes is also called insulin-dependent. It frequently occurs in adolescence and is mainly characterized by insufficient insulin secretion [4, 5]. Type 2 diabetes, also known as noninsulin-dependent diabetes, often occurs in adulthood. It is relatively rare in childhood and is mainly caused by the inability of the body to effectively use insulin [6]. Clinically, more than 90% of diabetic patients belong to type 2 diabetes. The causes of this type of diabetes are mostly lack of physical exercise and overweight [7, 8]. The clinical symptoms of type 2 diabetes are similar to those of type 1 diabetes, but the degree of manifestation is relatively mild, and the diagnosis is often not detected for several years. In most cases, the diagnosis of type 2 diabetes is due to the appearance of complications [9–12].

The article "High-Resolution Computer Tomography Image Features of Lungs for Patients with Type 2 Diabetes under the Faster-Region Recurrent Convolutional Neural Network Algorithm" was retracted in 2023. Reasons: signs of a paper mill; suspected computer-generated content; unreliable results or conclusions; concerns about the data.

Diabetic patients often have lung infections. According to research statistics, about 10% of diabetic patients die from infections, of which about one-third of deaths caused by lung infections [13, 14]. Many factors can cause lung infections in diabetic patients. When the blood sugar is at a high level, the patient's immune function will be impaired, which will lead to a lack of respiratory tract immunity, and a large number of bacteria will invade and cause lung infections. In addition, glycerol products increase in a large amount when the body is in a high-sugar state, providing nutrients for bacteria and causing infection; when the body is in a high-sugar state, the protein is decomposed in a large amount and the synthesis is reduced, resulting in insufficient immune molecules such as antibodies and complement, which cannot resist the invasion of pathogens, causing the pathogens to enter the lungs and multiply [15–19]. Pulmonary microvascular disease occurs in diabetic patients, capillary damage causes the reduction of the effective air exchange area of the alveoli, and the lack of oxygen in the lung tissue can easily lead to infection [20–22]. Diabetic patients reduce the synthesis of 2-3 diphosphate glycerol in the red blood cells and increase the glycated hemoglobin A1c (HbA1c) in the blood, so that the oxygen dissociation curve of hemoglobin shifts to the left, which is not conducive to the release of oxygen. The increase in growth hormone and other factors in the body is in a hypoxic state, which causes the blood sugar level to rise, increasing the risk of infection [23, 24]. In diabetic patients, the liver's ability to convert vitamin A is reduced, and the lack of vitamin A leads to slower airway epithelial repair, which causes abnormal secretion of respiratory mucosal cells and hyperkeratinization of the epithelium, and weakens the ability of lung tissue to resist bacteria [25–27].

The article "High-Resolution Computer Tomography Image Features of Lungs for Patients with Type 2 Diabetes under the Faster-Region Recurrent Convolutional Neural Network Algorithm" was retracted in 2023. Reasons: signs of a paper mill; suspected computer-generated content; unreliable results or conclusions; concerns about the data.

In recent years, with the rapid development of computer technology, deep neural network technology has made great progress in the field of image recognition. The faster-region convolutional neural network (Faster-RCNN) algorithm is widely used in medical imaging diagnosis. Based on the analysis of a large number of medical images and the extraction of image features, some researches build the Faster-RCNN intelligent recognition model, so as to achieve the goal of efficiently and accurately processing medical imaging data, and overcome the problem of different clinical doctors facing the same diagnostic difference in the same image, reducing the work intensity of imaging work physicians [28, 29]. At present, the Faster-RCNN algorithm has achieved satisfactory results in the identification of clinical image feature information of prostate cancer, lung cancer, and rectal lymph nodes [30, 31]. However, researchers still mainly focus on functional research and basic research on lung damage caused by diabetes [32]. There are few studies on the high-resolution computed tomography (HRCT) imaging of the diabetic lung. Compared with conventional CT, the application of HRCT in pulmonary lesions in patients with type 2 diabetes significantly improved the diagnostic performance. In addition, it can detect the shape of the lesion and display the density inside the lesion and the subtle features of the lesion edge, and its association of the adjacent blood vessels is more accurate, providing more detailed reference information for clinical diagnosis [33, 34]. In order to understand the morphological changes of the lung damage in diabetic patients, it is extremely important to study the HRCT imaging characteristics of the diabetic lung.

To use HRCT based on Faster-RCNN algorithm to evaluate various imaging features of lung lesions in patients with type 2 diabetes, 176 patients with type 2 diabetes were selected as the research objects, and they were divided into different groups based on gender, course of disease, age, glycosylated hemoglobin level (HbA1c), 2 h C peptide (2 h C-P) after meal, fasting C peptide (FC-P), and complications. The research objects were performed with HRCT scan, and the Faster-RCNN algorithm model was built to obtain the imaging features. The relationships between HRCT imaging features and 2 h C-P, FC-P, HbA1c, gender, course of disease, age, and complications were analyzed comprehensively, so as to evaluate the application value of the HRCT imaging features of the Faster-RCNN algorithm in the assessment of lung disease in patients with type 2 diabetes.

The article "High-Resolution Computer Tomography Image Features of Lungs for Patients with Type 2 Diabetes under the Faster-Region Recurrent Convolutional Neural Network Algorithm" was retracted in 2023. Reasons: signs of a paper mill; suspected computer-generated content; unreliable results or conclusions; concerns about the data.

## 2. Materials and Methods

### 2.1. Research Objects

In this study, 176 patients with type 2 diabetes in the hospital from February 2019 to September 2021 were selected as the research objects, and they were divided into different groups based on gender, course of disease, age, glycosylated hemoglobin level (HbA1c), 2 h C peptide (2 h C-P) after meal, fasting C peptide (FC-P), and complications. There were 89 males and 87 females. There were 62 cases with the course of disease less than 5 years, 58 cases with the course of disease of 6-10 years, and 56 cases with the course of disease of more than 10 years. They were rolled into three subgroups based on the age: 35-50-year-old group (57 cases), 51-65-year-old group (59 cases), and over 65-year-old group (60 cases). According to the HbA1c content, the patients can be rolled into an effective control (less than 7% (54 cases)), a general control group (7%-10% (65 cases)), and an ineffective control group (more than 10% (57 cases)). According to the different 2 h C-P values, the patients were rolled into four subgroups: less than 1.09 nmol/L group (45 cases), 1.1-1.48 nmol/L group (43 cases), 1.49-2.11 nmol/L group (44 cases), and more than 2.11 nmol/L (44 cases). In the term of FC-P, they were divided into less than 0.26 nmol/L group (45 cases), 0.27-0.45 nmol/L group (46 cases), 0.46-0.6 nmol/L group (42 cases), and more than 0.6 nmol/L group (43 cases). The patients could be grouped into 4 (group 0 (40 cases), group 1 (48 cases), group 2 (46 cases), and group 3 (42 cases)) according to whether the microvascular disease, nervous system disease, and diabetic foot occurred. The mean age of all patients was 60.23 ± 6.87, and the gender ratio of male patients to female patients was 89 : 87. This study had been approved by the Medical Ethics Committee of Hospital, and the family members of the patients had understood the research situation and signed the informed consent forms.

The following are the inclusion criteria: patients who were diagnosed as high type 2 diabetes according to the diabetes diagnosis and classification criteria given by the World Health Organization (WHO), patients with no acute metabolic disorders or disorders, patients without other serious organ damage diseases, and patients without examination contraindications.

The following are the exclusion criteria: patients with pulmonary diseases such as tuberculosis that may affect the results of this study, patients with a long-term smoking history, patients who were pregnant or breastfeeding, patients with primary heart or lung disease (pulmonary edema, heart failure, angina pectoris, myocardial infarction, etc.), and patients with mental illness.

The article "High-Resolution Computer Tomography Image Features of Lungs for Patients with Type 2 Diabetes under the Faster-Region Recurrent Convolutional Neural Network Algorithm" was retracted in 2023. Reasons: signs of a paper mill; suspected computer-generated content; unreliable results or conclusions; concerns about the data.

### 2.2. HRCT Imaging Scan

HRCT imaging examination was performed. The examination instrument used 64-slice spiral CT scanner. The patient was placed in the supine position and then the whole lung scan was performed. The patient lifted his hands up and held his breath after a deep inhalation to scan the whole lung: between the lungs to the base of the lungs. First, the whole lung was scanned, and after the lesions were found, local HRCT was performed on the lungs. For those who needed to consider the ground-glass shadow and the impact of gravity on the back, the prone position was scanned under the same scanning conditions. The specific conditions of the scan are shown in Figure 1. HRCT local scan was performed on the lesion to obtain a scanned image. Image acquisition is as follows: all image data in high resolution was sent to the workstation for postprocessing. The window width was between 1000 and 1600 HU, and the window level was adjusted as -650 to -750.

### 2.3. Faster-RCNN Algorithm

The Faster-RCNN algorithm model was mainly composed of six modules: input images and labels, convolutional layer, region of interest (ROI) pooling layer, region proposal network (RPN), fully connected layer, and classification regression module. The operation steps were as follows. After an image of any scale was inputted, it could enter the convolutional layer through adjustment to obtain the feature map of the image. RPN extracted the feature blocks of the candidate frame through the feature map, and the ROI pooling layer extracted the feature maps of the first two. It was sent to the fully connected layer, and then, the final classification and regression was performed. The specific module analysis is shown in Figure 2.

Faster-RCNN selected candidate frames through RPN. In order to make the selected candidate frame close to the calibrated target block, the corresponding mapping relationship needed to be found. The feature block of the candidate frame transmitted by RPN was named K, and the basic information of the candidate frame was expressed by its coordinates and width and height as (*K*_*x*_, *K*_*y*_, *K*_*w*_, *K*_*h*_), where *K*_*x*_, *K*_*y*_, *K*_*w*_, and *K*_*h*_ represent coordinate information and width and height information, respectively. In addition, the boxes corresponding to the calibration box and the mapping relationship were named B and R, respectively, and the relationship among the three types of boxes is shown in Figure 3.

The article "High-Resolution Computer Tomography Image Features of Lungs for Patients with Type 2 Diabetes under the Faster-Region Recurrent Convolutional Neural Network Algorithm" was retracted in 2023. Reasons: signs of a paper mill; suspected computer-generated content; unreliable results or conclusions; concerns about the data.

The basic information of the two boxes B and R was also displayed according to the coordinate position and width and height. This regression relationship was shown in

(1) $$\begin{array}{c} f\left(K_{x},K_{y,}K_{w},K_{h}\right)=\left(R_{x},R_{y,}R_{w},R_{h}\right)\approx \left(B_{x},B_{y,}B_{w},B_{h}\right). \end{array}$$

When the candidate frame output by RPN shifted, the horizontal and vertical coordinates in the basic information would change accordingly, as shown in

(2) $$\begin{array}{c} R_{x}=K_{x}+\nabla x=K_{x}+K_{w}d_{x}\left(K\right), \end{array}$$

(3) $$\begin{array}{c} R_{y}=K_{y}+\nabla y=K_{y}+K_{w}d_{y}\left(K\right). \end{array}$$

When the candidate frame output by RPN was scaled, the width and height in the basic information would change accordingly, as shown in

(4) $$\begin{array}{c} R_{w}=K_{w}e^{d_{w}\left(K\right)}, \end{array}$$

(5) $$\begin{array}{c} R_{h}=K_{h}e^{d_{h}\left(K\right)}. \end{array}$$

After panning and zooming, the coordinates and width and height information that were closest to the calibration frame were obtained as (*R*_*x*_, *R*_*y*_, *R*_*w*_, *R*_*h*_).

### 2.4. Evaluation Indicators

The internationally accepted method was adopted to quantify the HRCT features for scoring. Firstly, the lung visual field was divided into 12 areas through the tracheal carina and above, the right lower pulmonary vein and below, and the front and back half. According to the percentage of the area of the lung parenchymal lesions, the scoring level was determined, which was divided into the following six levels. 0 point meant no abnormality, 1 point meant the area was less than 1%, 2 points meant that the area accounted for 5%~25%, 3 points represented 26%-50% of the area, 4 points represented 51%-75% of the area, and 5 points represented an area greater than 75%. The scoring standard for the degree of bronchiectasis was as follows: 0 point meant 1-1.5 times the normal state when the diameter of the expanded bronchus was expanded, 1 point meant 1.5-2 times, and 2 points meant 2 times or more.

The lung HRCT imaging differences in different groups of diabetic patients were recorded and analyzed to determine whether HRCT imaging features were related to gender, course of disease, age, HbA1c, 2 h C-P, FC-P, and complications after a meal.

Three common indicators were selected to evaluate the effect of HRCT based on Faster-RCNN algorithm in diagnosing diabetic lung lesions: accuracy, specificity, and sensitivity. The calculation methods were

(6) $$\begin{array}{c} \text{Accuracy}=\frac{A+B}{A+C+B+D}, \end{array}$$

(7) $$\begin{array}{c} \text{Specificity}=\frac{B}{C+B}, \end{array}$$

(8) $$\begin{array}{c} \text{Sensitivity}=\frac{A}{D+A}. \end{array}$$

In the above equations, *A* referred to true positive, which meant that the diagnosis result was positive and actually was positive; *B* was true negative, which meant that the diagnosis result was negative but was actually negative; *C* (false positive) meant that the diagnosis result was positive, but the actual result was negative; *D* (false negative) meant that the actual result was positive and the diagnosis result was negative.

The article "High-Resolution Computer Tomography Image Features of Lungs for Patients with Type 2 Diabetes under the Faster-Region Recurrent Convolutional Neural Network Algorithm" was retracted in 2023. Reasons: signs of a paper mill; suspected computer-generated content; unreliable results or conclusions; concerns about the data.

The receiver operating curve (ROC) was used to express the diagnostic efficiency of HRCT based on the Faster-RCNN algorithm, the area under curve (AUC) was determined according to the ROC, and comparative analysis was performed.

### 2.5. Statistical Methods

The SPSS software was used to statistically analyze the data, and the data in accordance with the normal distribution were expressed as the mean ± standard deviation (mean ± S). The Wilcoxon rank-sum test was used for comparative analysis between groups, and the Spearman rank correlation was used to analyze the relationship between single factor and HRCT feature scores. *P* < 0.05 indicated that there was a statistical difference.

## 3. Results

### 3.1. HRCT Imaging Results of Type 2 Diabetic Patients

HRCT imaging examination was performed for type 2 diabetic patients with lung infection (as shown in Figure 4). It illustrated that the patient's lungs showed a variety of abnormal manifestations such as subpleural reticulation (Figure 4(c)), interstitial nodules (Figure 4(d)), thickening of interlobular septum and thickening of intralobular interstitial (Figure 4(e)), cellular lung (Figure 4(f)), bronchiectasis (Figure 4(g)), and peribronchial interstitial thickening (Figures 4(h) and 4(i)). Figures 4(a) and 4(b) were HRCT images of normal lungs.

### 3.2. The Relationship between Gender and Course of Disease of Patients and HRCT Score

The Wilcoxon rank-sum test was used to evaluate the relationship between gender and course of disease of patients and HRCT scores. The HRCT score in the male patient group was 3.76, and that in the female patient group was 3.81. It was found that there was no obvious difference in HRCT scores between male and female patients in the gender group (*P* > 0.05); in the course of disease group, the mean HRCT scores of the three groups of patients with different disease courses were 1.77, 3.92, and 5.23, respectively. The HRCT scores of patients with course of disease of 6-10 years and >10 years increased greatly compared with 0-5 years of course of disease patients (*P* < 0.05). The specific results are shown in Figure 5.

The article "High-Resolution Computer Tomography Image Features of Lungs for Patients with Type 2 Diabetes under the Faster-Region Recurrent Convolutional Neural Network Algorithm" was retracted in 2023. Reasons: signs of a paper mill; suspected computer-generated content; unreliable results or conclusions; concerns about the data.

The Spearman rank correlation analysis was adopted to assess the relationship between course of disease and HRCT score. The scatter plot results showed a positive correlation between the two, as illustrated in Figure 6.

### 3.3. The Relationship between Age and Complications of Patients and HRCT Score

The Wilcoxon rank-sum test was used to evaluate the relationship between age and complications of patients and HRCT score, as revealed in Figure 7. The mean HRCT scores of patients in different age groups were 3.45, 3.24, and 3.34, respectively. It was found that there was no observable difference in HRCT scores among patients of all age levels in the age group (*P* > 0.05). In the complications group, as the patients' complications score increased, the mean HRCT scores were 2.25, 3.98, 5.46, and 6.87, respectively, and the HRCT score increased greatly (*P* < 0.05).

The Spearman rank correlation analysis was adopted to assess the relationship between complications and HRCT scores. The scatter plot results showed that there was a positive correlation between the two. The specific results are shown in Figure 8.

### 3.4. The Relationship between HbA1c, 2 h C-P, and FC-P of Patients and HRCT Score

The Wilcoxon rank-sum test was used to evaluate the relationship between HbA1c, 2 h C-P, and FC-P of patients and HRCT score after a meal. The mean HRCT scores of the effective control group, the general control group, and the ineffective control group were 3.88, 3.95, and 3.99, respectively. It was found that there was no visible difference in HRCT scores between patients with different HbA1c content in the HbA1c group (*P* > 0.05); in the 2 h C-P and FC-P groups after a meal, the mean HRCT scores of patients in different groups were 5.68, 3.97, 2.68, and 1.43, respectively, and the mean HRCT scores of patients with different FC-P content were 5.67, 3.81, 2.92, and 1.74, respectively. Therefore, the HRCT score was significantly reduced with the increase in the content of 2 h C-P and FC-P after a meal (*P* < 0.05). The specific results are shown in Figure 9.

The Spearman rank correlation analysis was applied to assess the relationship between 2 h C-P and FC-P of patients and HRCT scores after a meal. The scatter plot results showed that there was a negative correlation between 2 h C-P and FC-P of patients and HRCT scores after a meal. The specific results are given in Figure 10.

### 3.5. Diagnostic Test Results of HRCT Images Based on Faster-RCNN Algorithm for Type 2 Diabetic Patients with Lung Infection

The accuracy, specificity, and sensitivity of HRCT image diagnosis of type 2 diabetes for patients with lung infection based on Faster-RCNN algorithm were calculated, which were 90.12%, 90.43%, and 83.64%, respectively. The ROC was drawn, and the AUC was calculated according to the ROC, which was 0.895. The result is shown in Figure 11.

The article "High-Resolution Computer Tomography Image Features of Lungs for Patients with Type 2 Diabetes under the Faster-Region Recurrent Convolutional Neural Network Algorithm" was retracted in 2023. Reasons: signs of a paper mill; suspected computer-generated content; unreliable results or conclusions; concerns about the data.

## 4. Discussion

At present, the aging of the population is becoming increasingly severe, and the people's living standards continue to improve. The incidence of diabetes in China is showing an increasing trend year by year. Among them, type 2 diabetic patients account for more than 90% of the total number of diabetes [35]. Diabetes has been called the three major types of diseases together with cardiovascular and cerebrovascular diseases and cancer. Diabetic patients often have immune dysfunction or damage, so it is very easy to cause coinfection. According to statistics, 10% of diabetic patients die from infection, especially lung infection; and the number of deaths caused by lung infection accounts for about one-third of the death toll [36]. As one of the common complications of diabetes, lung infection can cause severe hyperglycemia and metabolic disorders in patients, which is usually difficult to control [37]. In the current research, the lung damage to diabetes is still mainly in functional research and basic research, and there are few researches on high-resolution computer tomography HRCT imaging of the lungs of diabetes. In order to deeply understand the morphological changes of lung damage in diabetic patients, it is extremely important to study the HRCT imaging characteristics of diabetic lungs.

In this study, 176 patients with type 2 diabetes were selected as the research objects, and they were divided into different groups. The research objects were performed with HRCT scan, and the Faster-RCNN algorithm model was built to obtain the imaging features. The relationships between HRCT imaging features and 2 h C-P, FC-P, HbA1c, gender, course of disease, age, and complications were analyzed comprehensively. The results showed that the patient's lungs showed multiple HRCT images such as subpleural reticulation, interstitial nodules, thickening of interlobular septum, thickening of interlobular interstitium, honeycomb lung, bronchiectasis, and peribronchial interstitial thickening. The HRCT score of the male patient group was 3.76, and that of the female patient group was 3.81. The Wilcoxon rank-sum test showed that there was no obvious difference in HRCT scores between male and female patients in the gender group, and the mean HRCT scores of patients in different age groups were 3.45, 3.24, and 3.34, respectively, so there were no significant differences in HRCT scores between patients in all age levels in the age group. In addition, the mean HRCT scores of the effective control group, the general control group, and the ineffective control group were 3.88, 3.95, and 3.99, respectively. There was no significant difference in HRCT scores between patients with different HbA1c content in the HbA1c group (*P* > 0.05). In the course of disease group and the complications group, as the patients' course of disease and complications increased, their HRCT scores increased greatly (*P* < 0.05). In the 2 h C-P group and FC-P group after a meal, as the content of 2 h C-P and FC-P after the meal increased, the HRCT score was significantly reduced (*P* < 0.05). In addition, the Spearman rank correlation analysis results showed that course of disease and complications were positively correlated with HRCT scores, and 2 h C-P and FC-P levels after a meal were negatively correlated with HRCT scores. This suggested that clinically, HRCT imaging features can be used to evaluate lung infection in patients with type 2 diabetes and provide relevant reference information. ROC analysis results showed that the accuracy, specificity, and sensitivity of HRCT image diagnosis of lung infection of patients with type 2 diabetes based on Faster-RCNN algorithm were 90.12%, 90.43%, and 83.64%, respectively. According to the ROC, the AUC was 0.895. Diabetic peripheral neuropathy is a common complication of diabetes. The pulmonary interstitium includes a large number of connective tissues, blood vessels, and nerves, which are very important for the diagnosis of pulmonary lesions in diabetic patients. With the development of diagnosis and treatment technology and imaging, HRCT gradually surpasses conventional CT and plays an increasingly important role in diagnosis. Studies have shown that HRCT can display more comprehensive and detailed lung lesions. The Faster-RCNN model integrates feature extraction, classification, and regression into one network model, which speeds up detection and can effectively solve machine learning problems with large samples, and has been widely used [38]. Some studies use HRCT image features based on Faster-RCNN algorithm to diagnose pancreatic cancer. It is found that HRCT diagnosis is reproducible and can make accurate judgments. It is of great significance to the diagnosis and disease evaluation of early pancreatic cancer. Such results were in line with the results of this study [39]. In summary, the imaging features of HRCT based on the Faster-RCNN algorithm were related to a variety of clinical factors, which can provide a large amount of effective reference information for the diagnosis and evaluation of lung infection of patients with type 2 diabetes.

The article "High-Resolution Computer Tomography Image Features of Lungs for Patients with Type 2 Diabetes under the Faster-Region Recurrent Convolutional Neural Network Algorithm" was retracted in 2023. Reasons: signs of a paper mill; suspected computer-generated content; unreliable results or conclusions; concerns about the data.

## 5. Conclusion

In this study, 176 patients with hypertension were selected and divided into gender group, course of disease group, age group, HbA1c group, 2 h C-P group, FC-P group, and complications group. The HRCT scan was performed, and the Faster-RCNN algorithm model was built to obtain image features. In addition, the relationships of HRCT imaging features to 2 h C-P, FC-P, HbA1c, gender, course of disease, age, and complications of patients were analyzed. It was found that the HRCT scores of patients with type 2 diabetes with lung infection were not related to gender, age, and HbA1c content, but positively correlated with the course of disease and complications of patients, and negatively correlated with the 2 h C-P and FC-P content after a meal of patients. HRCT imaging features can provide effective information for the diagnosis and clinical evaluation of lung infection in patients with type 2 diabetes. The disadvantage of this study was that the source of the research objects was single, so it was not random and widely applicable. In subsequent research, analysis and research of multisite and multitype data samples would be considered, and the correlation between HRCT image features based on Faster-RCNN algorithm and type 2 diabetic lung infection would be further studied, aiming to provide more practical and credible reference basis for its application in early clinical diagnosis and disease evaluation.

## Figures and Tables

**Figure 1:** The specific conditions of the HRCT scan.

**Figure 2:** Framework of Faster-RCNN algorithm model.

**Figure 3:** Selection of Faster-RCNN candidate frame.

**Figure 4:** HRCT images of patients with type 2 diabetes with pulmonary infection.

**Figure 5:** Comparison on HRCT scores between gender group and course of disease group. Note: ∗ suggested the difference was statistically great (*P* < 0.05).

**Figure 6:** The relationship between course of disease and HRCT score.

**Figure 7:** Comparison on HRCT scores of patients in the age group and the complications group. Note: ∗ suggested the difference was statistically great (*P* < 0.05).

**Figure 8:** The relationship between complications and HRCT scores.

**Figure 9:** Comparison on HRCT scores of patients in HbA1c group, 2 h C-P group after meal, and FC-P group. Note: ∗ suggested the difference was statistically great (*P* < 0.05).

**Figure 10:** The relationship between 2 h C-P and FC-P after a meal to HRCT scores. Note: (a) was a scatter plot between 2 h C-P and HRCT scores after a meal; (b) was a scatter plot between FC-P and HRCT scores.

**Figure 11:** Diagnostic test and ROC curve results of HRCT images for type 2 diabetic patients with lung infection. Note: (a) showed the accuracy, specificity, and sensitivity of HRCT imaging in the diagnosis of lung infection of patients with type 2 diabetes; and (b) was the ROC of HRCT imaging for the diagnosis of lung infection of patients with type 2 diabetes.

The article "High-Resolution Computer Tomography Image Features of Lungs for Patients with Type 2 Diabetes under the Faster-Region Recurrent Convolutional Neural Network Algorithm" was retracted in 2023. Reasons: signs of a paper mill; suspected computer-generated content; unreliable results or conclusions; concerns about the data.

## Data Availability

The data used to support the findings of this study are available from the corresponding author upon request.
